# Raman Spectroscopy-Assisted Characterization of Nanoform MoS_2_ Thin Film Transistor

**DOI:** 10.1155/2022/3255615

**Published:** 2022-06-22

**Authors:** Rajasekaran Saminathan, Haitham Hadidi, Mohammed Tharwan, Ali Alnujaie, Jabril A. Khamaj, Gunasekaran Venugopal

**Affiliations:** ^1^Mechanical Engineering Department, Faculty of Engineering, Jazan University, P. O. Box 45142, Jazan, Saudi Arabia; ^2^Department of Materials Science, School of Technology, Central University of Tamil Nadu, Thiruvarur, 610005 Tamil Nadu, India

## Abstract

In this paper, we report the simple preparation and investigation of electrical transport properties of nanoform MoS_2_ thin film transistor (TFT) devices. MoS_2_ nanoparticles were synthesized by using the hydrothermal method. The physiochemical characterizations such as UV-vis, Fourier transform infrared, X-ray diffraction, and Raman spectroscopy studies were performed. Spin-coating was used to make the thin film on which silver electrodes were made. We observed nonlinear current-voltage (I-V) characteristics; however, the symmetricity was found in the I-V curve which confirms the no formation of the Schottky barrier between thin film and electrodes. Transistor transfer characteristics reveal that the TFT device is n-doped as more drain current modulation is observed when the positive gate voltage is applied. The relationship between gate-current and gate voltage studies concludes that there is no leakage gate current in the TFT device which further confirms the good reliability of transfer characteristics of a device. The device mobility was calculated as ~10.2 cm^2^/Vs, and the same was explained with plausible reason supported with Raman spectra analysis.

## 1. Introduction

Presently, two-dimensional materials (graphene, graphene-oxide, MoS_2_, and Bi_2_Se_3_) have been known for their unique characteristics and having potential prospects in various fields such as electronics, photovoltaic, sensors, flexible displays, supercapacitors, and water purification [1, 2]. Transition metal dichalcogenide semiconductors (TMDC) have significantly attracted the scientific community because of their unique electrical and optical characteristics. Molybdenum disulfide (MoS_2_) is a layered structure transition metal dichalcogenide material with weak van der Waals interlayer force, which is considered as a best candidate material for numerous applications such as supercapacitor, hydrogen generation/storage, photocatalyst, and rechargeable batteries [3–8]. MoS_2_ has a hexagonal atomic arrangement similar to graphene. Mo and S atoms are stacked together in a single lattice and the weak van der Waals forces exist between the interlayers. Monolayer or bulk MoS_2_ may have different functions due to bandgap. It has been reported that the bulk MoS_2_ having an indirect bandgap of 1.29 eV and monolayer MoS_2_ having a direct bandgap of 1.9 eV [9] exist in a few forms of crystal structures such as 1T-MoS_2_ (tetragonal), 2H-MoS_2_ (hexagonal), and 3R-MoS_2_ (rhombohedral) [10]. As per the report by Radisavljevic et al., the pristine single crystal-based MoS_2_ field effect transistors have shown mobility of 200 cm^2^/Vs with a current on/off ratio of 10^8^ [11]. Particularly, MoS_2_ received special attention among the TMDCs and believed as an alternative material for graphene (which has zero bandgap) in electronics [12].

By having salient features such as nominal bandgap, good carrier mobility, and interesting geometry, MoS_2_ rises as an important candidate material in electronics and transistor development [13]. MoS_2_ thin films have shown tremendous potentiality in the applications such as nanogenerators, electrochemical supercapacitors, photovoltaic cells, sensors, and detectors [14–16]. The thermal instability of nanomaterials is the unavoidable parameter for these devices, because the materials may be heated due to photon absorption, charge carrier flow, and surrounding environment which may affect the device performance. Substrate used for material deposition also plays a key role in thermal stability. Previously, it was reported that monolayer thin film on SiO_2_ substrate is thermally stable compared to bulk MoS_2_. However, the preparation of large area thin film with a uniform surface is still a quite difficult process and suitable appropriate methods have to be followed. Some reports were published recently on the large area thin films which were made using physical vapor deposition (PVD), chemical vapor deposition (CVD), vapor epitaxy, pulsed-laser depositor (PLD) and sputtering methods [14, 17]. These methods involve high costs and large manpower with complicated process procedures. Hence, a simple and cost-effective method is required as an alternative. In this work, we used a hydrothermal method to produce MoS_2_ nanoparticles and used spin-coating to make large area thin film. The hydrothermal method is a simple and cost-effective method through which good quality samples can be prepared and large area thin films can be formed by spin-coating with thickness control by standardizing the film-making procedures [18, 19].

In the recent past, only a few studies have been reported on the electrical transport properties of MoS_2_ thin film transistors (TFT) [20, 21], and their electronic transport properties and their mechanism are not explored well and required to be investigated more. Hence in this paper, we report the simple preparation procedure of MoS_2_ nanoparticles, thin film making, and the electrical transport characteristics of MoS_2_ TFT in detail.

## 2. Materials and Methods

### 2.1. Materials

All the research grade materials such as molybdenum oxide (MoO_3_), potassium thiocyanate, HCl (35 wt%), ethanol, and NaOH were purchased from Sigma-Aldrich and used without further purification. Deionized water is used in all experiments.

### 2.2. Preparation of MoS_2_ Samples

MoS_2_ nanoparticles were prepared by using the hydrothermal method [18, 22] using molybdenum oxide (MoO_3_) and potassium thiocyanate as precursor starting materials. Initially, 0.3 g of MoO_3_ (1.5 mmol) and 0.5 g of potassium thiocyanate (4 mmol) were dissolved in 50 mL of deionized water and the same was sonicated for 1 hr. Then, HCl solution (1 mol/L) was added in order to keep the solution pH value to 2.0, and the solution has been stirred for another 45 min. Thereafter, the solution has been transferred into a stainless-steel autoclave (Teflon-lined, 100 mL capacity) for the hydrothermal treatment at 250°C for 40 hrs. After the treatment, the system is allowed to be cooled to room temperature. Then, the centrifugation is done with 5000 rpm for 20 min resulting black colored MoS_2_ particles which were washed several times using ethanol and DI water. Then, the sample has been put inside a vacuum oven at 70°C (10 hrs) for drying. Spin-coating is used to prepare MoS_2_ thin film and silver paste was used to make contact electrodes.

### 2.3. Instrumentation

The absorption spectra of MoS_2_ nanoparticles were taken using the UV-vis spectrophotometer (model: Jasco V-670). Fourier transform infrared spectroscopy (FT-IR) was performed via FT spectrometer (model: Nicolet-6700, USA). Further, MoS_2_ thin film was analyzed with X-ray diffractometer (model: Shimadzu, XRD 6000) with Cu-K*_α_* radiation from the range of 10-70. Raman studies were done in Raman spectrometer (model: Horiba Scientific, LAbRAM). All the electrical transport analyses have been performed using the semiconductor parameter analyzer (model: Agilent, B1500A).

## 3. Results and Discussion

Surface morphology of MoS_2_ thin film has been studied by using scanning electron microscopy (SEM), transmission electron microscopy (TEM), and atomic force microscopy (AFM) techniques.

In Figure 1(a), the SEM image of MoS_2_ thin film is shown which clearly shows an irregular surface morphology of MoS_2_ thin film with wrinkled-like morphology. In Figure 1(b), the TEM image of MoS_2_ is shown which clearly depicts the sheet-like morphology with transparent nature. The 2D topography of MoS_2_ thin film was studied by using AFM ((which is shown in Figure 1(c)) which shows an average surface roughness of MoS_2_ thin film with value of 64 nm. This roughness is due to the overlapping of many MoS_2_ platelets so that the measured region might consist of overlapped MoS_2_ layers.

The optical image of MoS_2_ thin film is shown in Figure 2(a). The UV-vis spectroscopy graph as shown in Figure 2(b) reveals the absorption spectra at 208 nm. The peak observed in the near UV region is mainly caused by the excitonic characteristics of MoS_2_ nanoparticles [23]. In order to study the chemical compositions and vibration bonds in the sample, FT-IR measurement has been done which is shown in Figure 2(c). There is a feeble absorption peak at near 470 cm^−1^ which is ascribed to the characteristics Mo-S vibration mode and well-matched with the previous report [24].

The XRD pattern of the MoS_2_ thin film is shown in Figure 2(d). The main characteristic diffraction peak observed at 14.5° represents the (002) plane of the hexagonal structure of MoS_2_ and matched with the previous report [25]. Moreover, the other diffraction peaks were observed at 33°, 40°, 44°, 50°, and 61° representing the (100), (103), (005), (105), and (008) crystal planes of MoS_2_, respectively. This XRD data shows a good agreement with JCPDS card no. 37-1492.

### 3.1. Electrical Transport Studies

#### 3.1.1. Current-Voltage (I-V) Characterization of MoS_2_ Thin Film

The current-voltage characteristics of MoS_2_ thin film is shown in Figure 3(a).

It shows a slight nonlinear behavior. However, a clear symmetricity has been seen in I-V curve shown in Figure 3(b) which further confirms the no formation of the Schottky barrier between the contacts and thin film.

#### 3.1.2. Characterization of MoS_2_ Thin Film Transistor (TFT)

The schematic of the fabricated MoS_2_ TFT device is shown in Figure 4(a).

The transistor characteristics are studied for MoS_2_ thin film and their output characteristics (I_D_-V_DS_) for the different back-gate voltages (V_G_) varying from -25 to 25 V with a step of 10 V are shown in Figure 4(b). We observed a linear I_D_ versus V_DS_ curve, confirming an ohmic contact between thin film and electrodes. The transfer characteristics (I_D_-V_G_) of MoS_2_ TFT are shown in Figure 4(c), where the applied bias voltage is 100 mV.

When the gate voltage is increased, the drain current is also increased, which reveals the n-type behavior of TFT. Positive gate voltage produces more drain-current modulation than negative gate voltage (V_G_). The appearance of the charge neutrality point (V_CNP_) at the negative bias region (V_G_~-20 V) further concludes that the TFT device is n-doped.  Figure 5 shows the relationship between gate current (IG) and gate voltage (VG).

This shows the negligible gate current through the SiO_2_ oxide layer and confirms the excellent reliability of transfer characteristics presented in Figure 4(b). In addition, we extracted the mobility of our fabricated TFT device. The mobility (*μ*) of MoS_2_ TFT was calculated using the following.

(1) $$\begin{array}{c} \mu =\frac{L\times g_{m}}{W\times C_{ox}\times V_{d}}, \end{array}$$

where channel length (*L*) is equal to 30 *μ*m, the channel width (*W*) is equal to 25*μ*m, and the capacitance between the channel and back gate per unit area is *C*_ox_ where *C*_ox=_ *ξ*_0_ *ξ*_r_/*d* = 3.83 × 10^−8^ F/m^2^, where *ξ*_0_ is the permittivity of free space, *ξ*_r_ is 3.9 for SiO_2_, and *d* is gate oxide thickness (90 nm). We determined the mobility of MoS_2_ TFT as ~10.2 cm^2^/Vs from these data. This is comparable to the mobility of multilayer MoS_2_ transistor reported by Sharma et al. [26] where the mobility was reported as *μ*~15.3 cm^2^/V.s. The reduction in mobility is due to the defects that exist in the thin film which acts as scattering centers which resist the charge conduction. The reason for the low-mobility was further supported with Raman spectra analysis which is shown in Figure 6. The Raman spectra show two active modes at 381 cm^−1^ and 406 cm^−1^ which represent the E1_2g_ and A_1g_ vibration modes, respectively. Out of these two vibration modes, A_1g_ corresponds with the thickness of the layer and A_1g_ mode at 406 cm^−1^ reveals that the thin film may consist of several MoS_2_ sheets interlinked each other. As per the previous reports, the spin-coated thin films consist of several layers of MoS_2_ and its bulk counterpart [27, 28].

In general, the surface defects and structural disorders form traps in the form of wrinkles or folds on the surface, creating a small bulk counterpart in MoS_2_ thin film [29]. These traps are answerable for the observation of lower mobility in TFT devices. Breakage of S-Mo-S bonds during the synthesis process may lead to these kinds of traps/vacancy defects.

From the obtained results, we noticed that some sophisticated sample preparation techniques such as atomic layer deposition and chemical vapour deposition could be utilized to develop the high purity thin film for ultrafast response electronics devices.

## 4. Conclusion

The electrical transport characteristics of nanoform MoS2 thin film transistor device were investigated. MoS_2_ nanoparticles were prepared using the hydrothermal method. The as-prepared MoS_2_ samples were characterized with UV-vis, FT-IR, and X-ray diffraction techniques. Back-gated MoS_2_ transistor device was made with silver electrodes as a source and drain. The current-voltage characteristics show a nonlinear behaviour. But the observation of symmetricity in the I-V curves confirms the nonexistence of the Schottky contact between the thin film and contacts. Transistor characteristic studies further reveal that the TFT device is n-doped while registering the charge neutrality point at the negative bias region. The relationship between gate current and gate voltage with zero gate current shows the good solidarity of transfer characteristic results. The device mobility is calculated as ~10.2 cm^2^/Vs, which has a well agreement with the data reported for the MoS_2_ transistor. The observation of lower mobility in our MoS_2_ TFT device is further plausibly explained with Raman spectra analysis.

## Figures and Tables

**Figure 1:** (a) SEM image of MoS_2_ thin film. (b) TEM image of MoS_2_ nanofilm. (c) AFM image of MoS_2_ thin film, showing the thickness profile of 64 nm.

**Figure 2:** (a) Optical photograph of MoS_2_ thin film. (b) UV-vis spectra of MoS_2_ nanoparticles. (c) FT-IR spectra of MoS_2_ nanoparticles. (d) XRD spectra of MoS_2_ thin film.

**Figure 3:** (a) Current-voltage characteristics of MoS_2_ thin film. (b) Semilog I-V plot reveals a clear symmetricity.

**Figure 4:** (a) The schematic of the MoS_2_ TFT device. (b) Output characteristics (I_D_ versus V_DS_) of MoS_2_ TFT device at different back gate voltages. An apparent linear ohmic behavior is observed. (c) Transfer characteristics (I_D_-V_G_) of the same device.

**Figure 5:** Gate leakage current versus gate bias voltage characteristics of MoS_2_ TFT.

**Figure 6:** Raman spectra of MoS_2_ thin film.

## Data Availability

The complete data required for the representations are fully included in the research paper.
